The article "Bone-targeting drug delivery system of biomineral-binding liposomes loaded with icariin enhances the treatment for osteoporosis" was retracted in 2025. Reasons: errors in the images; unreliable data; concerns about the images.

# Bone-targeting drug delivery system of biomineral-binding liposomes loaded with icariin enhances the treatment for osteoporosis

**DOI:** 10.1186/s12951-019-0447-5

**Published:** 2019-01-22

**Authors:** Xiaoduan Sun, Jun Wei, Jiayao Lyu, Tierong Bian, Zhongbing Liu, Juan Huang, Fengjuan Pi, Chunhong Li, Zhirong Zhong

**Affiliations:** 1 Department of Pharmaceutical Sciences, School of Pharmacy, Southwest Medical University, Luzhou, 646000 Sichuan China; 2 Luzhou TCM Hospital, Luzhou, 646000 Sichuan China; 3 Medical Experimental Center, The Affiliated Hospital of Southwest Medical University, Luzhou, 646000 Sichuan China; 4 Department of Pharmacy, The Affiliated Hospital of Southwest Medical University, Luzhou, 646000 Sichuan China; 5 Key Laboratory of Medical Electrophysiology, Ministry of Education, Institute of Cardiovascular Research of Southwest Medical University, Luzhou, 646000 China

**Keywords:** Liposomes, Osteoporosis, Icariin, Hydroxyapatite, Pyrophosphate

## Abstract

**Background:**

Osteoporosis is a bone-incapacitating malady and it is characterized by obvious bone mass loss and bone microarchitecture deterioration. Current treatments for osteoporosis have many limitations, including the non-obvious therapeutic effect and long-term safety issues. Icariin is a pharmacologically active flavonoid glycoside, which shows potential application in treatment of osteoporosis. But its clinical application is limited by the inherent disadvantages such as poor water solubility, first pass effect after oral administration, and low bioavailability. Moreover, due to lack of targeting ability, icariin cannot accumulate at the local diseased region to provide early protection from fractures. To solve the application problems of icariin and enhance its therapeutic effects on osteoporosis, this work aimed to design a targeting drug delivery system of biomineral-binding liposomes (BBL) mediated by pyrophosphate ions.

**Results:**

Biomineral-binding liposomes enhanced the binding ability of liposomes with hydroxyapatite particles. It increased the serum level of alkaline phosphatase and reduced that of tartrate-resistant acid phosphatase 5b. Meanwhile, BBL increased the mechanical strength of femoral midshaft, preserving the trabecular bone microarchitecture. Moreover, BBL could initiate bone turnover/remodeling of rats with osteoporosis.

**Conclusions:**

This drug targeting delivery system of BBL loading with icariin showed more therapeutic advantages than the free icariin for the treatment of osteoporosis, which may be a kind of valid candidate in future osteoporosis therapy.

**Electronic supplementary material:**

The online version of this article (10.1186/s12951-019-0447-5) contains supplementary material, which is available to authorized users.

## Background

Osteoporosis is a typical age-related disease and it is more common in female than in male. Osteoporosis affects about half of the over-75-year-old female [1]. Osteoporosis is characterized by fragile bones and microarchitectural deterioration, which causes approximately 9 million cases of the bone fractures every year [2].

Current clinical treatments on osteoporosis mainly include estrogen therapy, bisphosphonates, and selective estrogen receptor modulators [3]. But these treatments showed obvious restrictions, including non-obvious therapeutic effect and long-term safety issues. For example, bisphosphonates were widely used for osteoporosis therapeutics, which avoided further bone deterioration in osteoporosis. But, it can’t replenish the already lost bone [3, 4]. What’s more, oral bisphosphonates may cause esophageal irritation and the intravenous injection of bisphosphonates with rapid speed may cause renal toxicity [3]. Estrogen therapy showed some non-skeletal adverse consequences such as breast carcinoma and vascular events [3]. Some other pharmacological treatments for osteoporosis include growth factors, calcium and vitamin D supplementation, calcitonin, and parathyroid hormone. Among them, treatment with calcium plus vitamin D supplementation for osteoporosis is controversial [5, 6]. It was reported that calcitonin can induce vascular symptoms and gastrointestinal symptoms [7, 8], and parathyroid hormone may cause life-threatening hypercalcemia [9]. Therefore, more candidates for osteoporosis need to be investigated in the basic research.

Icariin (C_33_H_40_O_15_, MW 676.65) is a kind of flavonoid glycoside extracted from the Chinese traditional medicine of Herba Epimedii. It has been reported that icariin could help with the treatment of osteoporosis [10]. Compared with the drugs mentioned above, icariin focuses on the maturation of osteoblasts [11]. It improves the activity of alkaline phosphatase (ALP) and increases the expression of receptor activator of nuclear factor κ-B ligand to promote the bone formation [11]. It also affects the bone morphogenic protein-2 (BMP-2)/Smad4 pathway thus up regulates the expression of BMP-2 and Smad4, resulting in the formation of calcified nodules in bone [11]. Icariin also leads to G2/M block,which decreases the bone resorption and attenuates the expression of tartrate-resistant acid phosphatase (TRACP) by osteoclasts thereby accelerating the accumulation of trace elements such as calcium and phosphorus in bones and improving osteoporosis [11]. Icariin has been widely used in orthopedic practice, and many of its therapeutic effects on bone problem and fractures have been reported [12, 13]. Moreover, icariin is more effective in promoting osteogenic differentiation than other natural flavonoids like genistein [11]. Meanwhile, icariin is a botanical compound that can stimulate increased sex hormone levels and interact with the estrogen receptor to produce hormone-like action [14]. But the inherent disadvantages of icariin such as poor water-solubility, first pass effect after oral administration, and low bioavailability limited the clinical applications. Moreover, due to lack of targeting ability, icariin cannot accumulate at the local diseased region to provide early protection from fractures.

Among the nano-sized drug delivery carriers, liposomes were widely used, having good biocompatibility and controlled release ability [15, 16]. Currently, liposomes, such as paclitaxel liposomes and doxorubicin liposomes, have been used in clinical therapy [17]. Liposome composed of phospholipid is a kind of spherical vesicle with lipid bilayer. The phospholipid is composed of hydrophilic heads and hydrophobic tails which formed a self-assembled nanostructure through hydrophobic interactions [18]. The hydrophilic cargos can be wrapped in the aqueous core while the hydrophobic drugs were kept in the lipid bilayer of liposomes [19]. On the other hand, it was reported that an alendronate-tri(ethyleneglycol)-cholesterol (ALN-TEG-Chol) conjugate showed rapid and strong binding ability to hydroxyapatite (HA) [20]. With other excipients, ALN-TEG-Chol was used to prepare biomineral-binding liposomes (BBL) showing rapid and strong binding ability with HA. The same concept can be extrapolated easily to other targeting moieties, e.g. tris (tetra-*n*-butylammonium) hydrogen pyrophosphate as a specific binding moiety to the same surface has been developed.

Based on these reports, we designed and synthesized a novel pyrophosphate-tri (ethyleneglycol)-cholesterol conjugate (PPi-TEG-Chol), taking pyrophosphate (PPi) as the targeting part with strong affinity with bone [21]. We hypothesized that as shown in the schematic diagram (Fig. 1), designing a targeting drug delivery system of BBL mediated by PPi could solve the application problems of icariin and enhance its therapeutic effects on osteoporosis. It may form novel liposomal delivery platform, which would provide novel therapeutic approach for the treatment of osteoporosis by anchoring to HA surface and gradually releasing icariin.

**Fig. 1:** Schematic diagram about the bone-targeting drug delivery system of biomineral-binding liposomes (BBL) loaded with icariin enhancing the treatment of osteoporosis

Since HA is a main mineral constituent of bone, we investigated the in vitro targeting ability of BBL via the binding experiment of BBL with HA. The in vivo therapeutic effect of BBL taking non-binding liposome (NBL) as control was evaluated on the osteoporosis animal model constructed by ovariectomy (OVX) plus glucocorticoid (GLU) injection. We detected the bone formation marker of ALP and bone resorption marker of TRACP 5b by ELISA. Meanwhile, the mechanical strength and bone microstructure were evaluated respectively by a three-point bending test and a micro-computerized tomography (Micro-CT) analysis. We also carried out histological studies including TRACP staining, Alizarin red staining, and hematoxylin and eosin (H&E) staining.

## Results

### Characterization of BBL preparations

The trans-mission electron microscopy (TEM) detection demonstrated that both BBL and NBL showed a uniform spherical shape (Fig. 2a–f). Results from the dynamic light scattering (DLS) detection (Table 1) showed that BBL and NBL had an average particle size of 193.10 ± 0.80 nm and 152.30 ± 0.70 nm, with a zeta potential of − 5.53 ± 0.10 mV and − 1.30 ± 0.20 mV, respectively. The polydispersity index (PDI) resulted from BBL and NBL is 0.19 ± 0.01 and 0.24 ± 0.01, respectively. It suggested that these liposomes might have a narrow size distribution, which was confirmed by the results shown in Fig. 2g, h. Results from HPLC analysis indicated that icariin was incorporated into BBL with a remarkably high encapsulation efficiency of 87.40 ± 3.70%, and a drug loading yield of 4.30 ± 0.67%. Additionally, the retention time of icariin peak in BBL was consistent with that of standard icariin. No interference peaks were observed in the near location of icariin peak. The result indicated that this HPLC method developed in this study was sensitive enough to determine icariin. In terms of the linearity, the result demonstrated that the standard curve was linear over the range of 180–1650 μg/mL with an excellent correlation between peak area and concentration of icariin (A = 1447C + 47.13, R^2^ = 0.9966). The results of the accuracy and precision demonstrated that the analysis method established in this study showed the intra- and inter-day relative standard deviation (RSD) was less than 10% for these samples. The extraction recoveries of icariin at low, medium and high concentration levels were 99.79 ± 0.38% (RSD, 0.38%), 100.61 ± 0.90% (RSD, 0.89%), and 100.17 ± 0.72% (RSD, 0.72%), respectively. All the results suggested that the encapsulation efficiency was reliable under the established analysis method.

**Fig. 2:** Characterization of liposomes. Morphology detection of NBL (**a**, **c**, **e**) and BBL (**b**, **d**, **f**) by TEM detection, and the size distribution of NBL (**g**) and BBL (**h**) by a method of DLS. The bar is 1 μm in (**a**, **b**), 200 nm in (**c**, **d**), and 100 nm in (**e**, **f**)

**Table 1:** Composition and characterization of liposomes

Liposomes	Molar ratios (A/B/C)	Particle size (nm)	PDI	Zeta potential (mV)	Drug loading (%)	Encapsulation efficiency (%)
NBL	70/30/0	152.3 ± 0.7	0.24 ± 0.01	− 1.3 ± 0.2	3.8 ± 0.83	78.6 ± 4.9
BBL	70/20/10	193.1 ± 0.8	0.19 ± 0.01	− 5.53 ± 0.1	4.3 ± 0.67	87.4 ± 3.7

Values were expressed as the mean ± S.D. from three independent experiments

A: Soybean lecithin; B: cholesterol; C: PPi-TEG-Chol; NBL: non-binding liposomes; BBL: biomineral-binding liposomes; PDI: polydispersity index

### BBL enhancing the binding potential and kinetics with HA particles

As shown in Fig. 3, after incubation for 30 min with the commercial synthetic HA (Fig. 3A) or the biotechnical HA (Fig. 3B), both free fluorescein sodium (Fig. 3A(a), B(a)) and BBL (Fig. 3A(c), B(c)) groups showed nearly no fluorescence, and fluor-NBL (Fig. 3A(b), B(b)) just showed very slight fluorescence. However, a very strong fluorescence was observed in the group of fluor-BBL (Fig. 3A(d), B(d)), in which the biotechnical HA particles showed stronger affinity with fluor-BBL than the synthetic HA did. These results may be due to the reason that PPi-TEG-Chol enhanced the binding ability of liposomes with HA particles.

**Fig. 3:** Biomineral-binding ability of liposomes with the commercial synthetic HA (**A**) and the biotechnical HA (**B**). The commercial synthetic HA and the biotechnical HA were separately incubated with fluorescein sodium (a), fluor-NBL (b), BBL (c) and fluor-BBL (d). It was observed under an AMG microscope with an EVOS^®^ XL fluorescence microscopy illumination system (40×). The quantitative detection of binding ability (**C**, **D**) was conducted by detecting the binded icariin through HPLC method. All data are shown as means ± standard deviations (n = 3)

In the binding kinetics study (Fig. 3C, D) measured by HPLC method, most of BBL loaded with icariin could swiftly bind to the biotechnical HA particles within 5 min and reached a binding plateau after 10 min with a binding rate of 75%. In the absence of PPi-TEG-Chol, NBL demonstrated a very limited non-specific binding to HA particles (< 15%). As for the commercial synthetic HA, the result of binding kinetics is similar except that the binding plateau of BBL and NBL is respectively about 50% and 15%, which indicated that for the same kind of liposomes, the biotechnical HA particles showed stronger affinity than the synthetic HA did. Meanwhile, PPi-TEG-Chol enhanced the binding ability of liposomes with HA particles.

### BBL showing a sustained-release profile

The in vitro release profile of icariin from liposomes was evaluated over a 100-h period. As shown in Fig. 4, the accumulative release rates was ~ 82% for free icariin and 50–60% for BBL or NBL at 10 h. Afterward, both BBL and NBL kept releasing continuously. The accumulative release rates of icariin from BBL and NBL at 96 h were 69.90 ± 2.21% and 80.60 ± 1.40%, respectively. These results suggested that both BBL and NBL showed good sustained release effect. This result is also consistent with that from in vivo pharmacokinetics evaluation in rats shown in Additional file 1: Fig. S1 and Table S1, in which the half-life of icariin, BBL and NBL is 3.3 h, 53.9 h and 38.2 h, respectively.

**Fig. 4:** In vitro release profile of icariin, BBL and NBL. The accumulative release of icariin from free icariin, BBL and NBL was conducted in PBS medium (pH 7.4) containing 0.3% Tween-80 at 37 °C. Results are presented as mean ± SD (n = 3)

### Detection of ALP and TRACP 5b in serum of rats

To access the treatment effects of BBL on the bone formation and bone resorption, we detected the serum levels of both ALP and TRACP 5b by ELISA method. As shown in Fig. 5a, the serum level of ALP showed no difference between NBL vs. FD (free drug) and SHAM (sham-control surgery) vs. BBL. In the BBL group, it was 20.40 ± 4.10 U/L which was the highest one among all the treatment groups; while in PBS group, it was 6.60 ± 0.40 U/L which was significantly lower than those in the other five treatments. Both FD group (11.80 ± 2.60 U/L) and NBL group (12.10 ± 1.80 U/L) showed significantly higher serum levels of ALP than PBS group (P < 0.05) after the treatments. The serum levels of TRACP 5b resulted from rats after treatment with the different formulation were presented in Fig. 5b. Compared to BBL group with a TRAP 5b level of 7.80 ± 0.80 U/L, FD and NBL remarkably increased it to 11.70 ± 0.50 U/L and 12.30 ± 0.50 U/L, respectively (P < 0.01). No significant difference was found in serum level of TRACP 5b between PBS and EBBL (empty biomineral-binding liposomes), FD and NBL. These results suggested that BBL could stimulate bone formation and suppress the bone resorption as well.

**Fig. 5:** Effects of different treatments on the bone formation marker of ALP (**a**) and the bone resorption marker of TRACP 5b (**b**). SD rats subjected to SHAM or to OVX combined with GLU injection were treated with PBS control (PBS), EBBL, NBL, FD and BBL, respectively. After 7 weeks post administration, serum was collected to detect both ALP and TRACP 5b by ELISA. Values are expressed as mean ± standard deviation (*P < 0.05, **P < 0.01)

### BBL enhancing the bone mechanical strength of rats subjected to OVX plus GLU

Results about the mechanical properties of femur via three-point bending tests were shown in Fig. 6. They indicated that the construction of osteoporosis model by OVX plus GLU brought on a significant reduction in the strength parameters including peak load, ultimate stiffness, ultimate strength and Young’s modulus.

**Fig. 6:** Effects of different treatments on the femoral biomechanical properties including peak load (**a**), ultimate stiffness (**b**), ultimate strength (**c**) and Young’s modulus (**d**). SD rats subjected to SHAM or OVX combined with GLU injection were treated with PBS control, EBBL, NBL, FD and BBL, respectively. Necks of left femora were subjected to the mechanical three-point bending test via a biomechanical testing system (MTS 858 Mini Bionix II, MTS Systems Corp., Eden Prairie, MN). Values are expressed as mean ± standard deviation (*P < 0.05, **P < 0.01, ***P < 0.001)

The peak load values of femur in the groups of NBL, FD, and BBL were 182.50 ± 12.70 N, 206.00 ± 8.20 N, and 262.10 ± 26.80 N, respectively, which were significantly higher than that in the PBS group with a value of 129.60 ± 13.90 N (P < 0.01, P < 0.01 and P < 0.05).

As for the ultimate stiffness of femur, the value resulted from PBS group was 348.30 ± 30.20 N/mm; but in the groups of NBL, FD, and BBL, it remarkably increased to 430.20 ± 29.90 N/mm, 506.90 ± 22.10 N/mm, and 623.80 ± 25.60 N/mm, respectively.

A similar increasing trend was observed in the ultimate strength of femur. The values from PBS, NBL, FD, and BBL was 34.40 ± 3.20 MPa, 43.70 ± 1.40 MPa, 44.20 ± 3.50 MPa and 60.70 ± 0.60 MPa, respectively.

The Young’s modulus values of femur in NBL (754.80 ± 96.10 MPa), FD (777.30 ± 17.30 MPa) and BBL (935.90 ± 26.20 MPa) were also significantly higher than that in the PBS group (505.20 ± 60.20 MPa).

Moreover, among all the strength parameters of peak load, ultimate stiffness, ultimate strength and Young’s modulus, there were no differences between the treatments of PBS vs. EBBL and SHAM vs. BBL; the values in FD group were significantly lower than that in BBL group. These results suggested that BBL loaded with icariin could significantly enhance the bone mechanical strength of rats subjected to the operation of OVX plus GLU.

### BBL contributing to restore the bone microarchitecture of rats with osteoporosis symptoms

The three-dimensional and two-dimensional reconstruction images of the TB microstructure resulted from Micro-CT assay are shown in Fig. 7a(I, II), respectively. The related quantitative analysis including the bone volume per tissue volume (BV/TV), bone surface per bone volume (BS/BV), trabecular thickness (Tb.Th), trabecular number (Tb.N), trabecular separation (Tb.Sp), and bone mineral density (BMD) were shown in Fig. 7b–g. The results showed that in PBS group, the parameter values of BV/TV, BS/BV, Tb.Th, Tb.N, Tb.Sp and BMD was 0.123 ± 0.005%, 56.390 ± 3.380 mm^−1^, 0.037 ± 0.002 mm, 3.090 ± 0.430 mm^−1^, 0.294 ± 0.043 mm, 243.920 ± 61.470 mg/cm^3^, respectively, which had significant differences compared to the corresponding parameter in the SHAM group with a value of 0.353 ± 0.013%, 32.430 ± 2.440 mm^−1^, 0.062 ± 0.004 mm, 9.230 ± 3.700 mm^−1^, 0.077 ± 0.005 mm, 966.360 ± 74.870 mg/cm^3^. For all the parameters, there was no difference between NBL and FD, PBS and EBBL, which suggested that EBBL might have no therapeutic effects on the rats subjected to surgery of OVX plus the injection of GLU. In BBL group, values of BV/TV, BS/BV, Tb.Th, Tb.N, Tb.Sp and BMD were 0.335 ± 0.011%, 34.370 ± 1.820 mm^−1^, 0.055 ± 0.002 mm, 8.410 ± 1.240 mm^−1^, 0.112 ± 0.008 mm, 786.080 ± 23.390 mg/cm^3^, respectively; while in FD group, they were 0.192 ± 0.008%, 37.950 ± 0.190 mm^−1^, 0.051 ± 0.001 mm, 5.020 ± 0.210 mm^−1^, 0.189 ± 0.005 mm, 588.970 ± 62.090 mg/cm^3^, respectively. And in NBL group, they were 0.185 ± 0.002%, 40.120 ± 0.580 mm^−1^, 0.049 ± 0.001 mm, 4.450 ± 0.320 mm^−1^, 0.214 ± 0.007 mm, 547.870 ± 23.420 mg/cm^3^, respectively. Statistical comparisons indicated that BBL treatment showed remarkable differences compared to FD or NBL treatments. These results indicated that BBL was helpful to restore the bone microarchitecture of rats with osteoporosis symptoms.

**Fig. 7:** Effects of various treatments on trabecular bone microarchitecture. SD rats subjected to SHAM or OVX plus GLU injection were treated with PBS control, EBBL, NBL, FD and BBL, respectively. The right femora of rats (n = 6) were analyzed by a high-resolution Micro-CT machine (SIMENS healthcare, Berlin and Munich, Germany) to get 3-dimensional Micro-CT images of the trabecular bone microarchitecture (**a**, I) and 2-dimensional Micro-CT images (**a**, II) of femoral necks. The quantitative characterization index, including BV/TV (**b**), BS/BV (**c**), Tb.Th (**d**), Tb.N (**e**), Tb.Sp (**f**) and trabecular BMD (**g**) were analyzed by Micro View software. Values are expressed as mean ± standard deviation (*P < 0.05, **P < 0.01)

### BBL promoting the bone remodeling process in osteoporosis rats according to histological results

The representative images from the histological analysis in the six groups via the H&E staining, TRACP staining and Alizarin red staining were shown in Fig. 8. The H&E staining of trabecular bone volume (TB, blue dotted area) in distal femora (Fig. 8a, d) showed that the TB volume in PBS group (0.18 ± 0.02) was significantly lower than those in control groups post drug injection (P < 0.05). Accordingly, a significantly higher TB volume was observed in BBL (0.55 ± 0.03) group compared with FD (0.32 ± 0.01) and NBL (0.26 ± 0.01) groups (P < 0.01 and P < 0.001, respectively). Interestingly, a significantly higher TB volume was observed in FD group as compared to NBL group (P < 0.01). In order to show the capability of osteoclastic resorption among the six groups during bone remodeling, TRACP staining was performed (Fig. 8b, e). In PBS group, osteoclasts in shuttle shape were observed, lining the osteoporotic trabecular surface. It was also found that a large number of mononuclear macrophages gradually fused and differentiated into mature osteoclasts (nuclei of TRACP positive staining cells ≥ 3). The least number of TRACP-positive cells with mature morphology was found in BBL group (2.57 ± 0.31) compared to the FD (5.64 ± 0.85) and NBL (6.52 ± 0.86) groups (P < 0.01 and P < 0.01, respectively). Alizarin red staining results (Fig. 8c, f) showed that PBS group (19.74 ± 3.30) exhibited lower cancellous bone mineralization rate compared to all other treatments (P < 0.05). Significantly increase of mineralization rate was found in BBL (56.65 ± 3.12) group post administration as compared with FD (32.49 ± 1.11) and NBL (25.76 ± 1.55) groups (P < 0.001 and P < 0.001, respectively). Likewise, a significantly higher mineralization rate was observed for FD group as compared to NBL group (P < 0.01). No significant difference was found between PBS and EBBL groups throughout the experimental period. These results demonstrated an activated bone remodeling process in osteoporosis rats treated with BBL.

**Fig. 8:** Effects of different treatments on the TB histomorphometry. SD rats subjected to SHAM or OVX plus GLU injection were treated with PBS control, EBBL, NBL, FD and BBL, respectively. The femoral necks were subjected to H&E staining (**a**), TRACP staining (**b**), and alizarin red staining (**c**), respectively. The quantitative analysis about the dynamic histomorphometric parameters of TB containing trabecular area ratio (**d**), proportion of positive osteoclast cells (**e**) and mineralized nodule proportion (**f**) was conducted. Values are expressed as mean ± standard deviation (**P < 0.01, ***P < 0.001)

## Discussion

Osteoporosis is one of the most common diseases of the elderly characterized by imbalance of bone formation and bone resorption, resulting in the deterioration of bone microarchitecture, low bone density, and poor bone strength [22]. In consideration of the limitation of systemic therapies, this study constructed a targeting drug delivery system for osteoporosis as the following steps. We synthesized the key component of BBL, pyrophosphate-tri(ethyleneglycol)-cholesterol (PPi-TEG-Chol), by chemical process for preparing BBL. Because of the high affinity of PPi with HA [20, 21, 23] crystals which is the major inorganic components in bones [24, 25], we chose it as the targeting moiety and conjugate it with cholesterol to form PPi-TEG-Chol, in which cholesterol was chosen as the molecule to introduce the bone-binding moiety due to its major role in the liposome lipid bilayer and a single secondary hydroxyl group in its structure facilitates chemical modification [26]. Moreover, both PPi and its major predictable metabolic product (i.e. phosphate) are considered as Generally Regarded As Safe (GRAS) by the FDA [27]. Liposomal formulation was chosen as our working platform owing to its long proven biocompatibility, versatility and the great potential of clinical translation [28, 29]. From the data generated by DLS analysis, BBL was found to be bigger than NBL in particle size and size distribution (193.1 nm and 152.3 nm), pointing out the addition of PPi-TEG-Chol did enlarge the particle size of the liposome formulation which may be due to the longer chain of PPi-TEG-Chol than that of single molecular of cholesterol.

We prepared the biotechnical HA under the conditions that are consistent with the bone biomineralization, taking the SIS membrane as the biomineralization template. In the biomineralization process of SIS, it is very important to ensure that the upper liquid would not leak from the edges and the SIS membrane would remain immersed into the liquid during the experimental period. The ions, Ca^2+^ and (HPO_4_)^2−^, diffused from the separate sides of SIS membrane and combined together to form the precipitate on some localized zones of SIS where there is a enough excessive saturation of Ca^2+^, (HPO_4_)^2−^ and OH^−^. As a result of the particular lower nucleation activation energy of SIS membrane towards the inorganic species, inorganic phases were prior to nucleation and emerged. After that, inorganic phase became larger along vertical direction of SIS film and it was oriented by the aligned collagen fibers of SIS. Above all, the procedure was growth of crystal cell of single-crystal flower-like HA, then growth plate-like HA rods. The size and structure of HA was regulated by SIS biotemplate. Growth direction of HA was perpendicular to SIS membrane. Because the manufacturing process and mechanism of HA resembled to that of the natural bones, the biotechnical HA is important in the long-term bone regeneration [30, 31]. It was reported that HA crystal belonged to the hexagonal system and classified into a(b)-plane HA and c-plane HA, in which the a(b)-plane HA is mainly positively charged calcium ions, and the c-plane HA is mainly negatively charged phosphate ions and hydroxyl groups. On the surface of long bone of amniotes, HA crystals possess a c-axis direction, which cause the growth of the a(b)-plane [32]. We synthesized the c-axis orientation HA according to our previous report [33], which caused the growth of the a(b)-plane and thus provided plenty of positive binding site for the negatively-charged PPi-TEG-Chol, showing a strong binding affinity. Meanwhile, although there is no PPi-TEG-Chol in the component of NBL, on the surface of NBL there is a very small amount of negative charges. Therefore, fluor-NBL groups could also show slight fluorescencein in the binding-ability detection.

We took the combination injection of OVX and GLU to establish osteopenia model in rats [34, 35], which showed evident decrease of bone formation, as proved by the reduced concentrations of serum ALP and BMD. These outcomes were accordance with some former findings by Jing et al. [36]. Treating the osteoporosis rats with the novel liposomal formulation provided a local drug (bone anabolic/anti-catabolic reagents) releasing to increase the bone formation and decrease the bone resorption. Serum ALP, an index of bone formation, was significantly lower in PBS group than that in SHAM group. BBL group was statistically superior to both FD and NBL groups in increasing the serum ALP of the OVX + GLU rats. OVX combined with GLU injection increased the serum concentration of TRACP 5b, which was a sensitive marker of bone resorption. Treatment with BBL was statistically superior to other therapeutic interventions in inhibiting the raise of serum TRACP 5b. Cortical bone played a key role in bone strength and the bone density and mechanical properties were linearly correlated [37]. In this research, the mechanical characteristics of rat femora declined in PBS group when compared to SHAM group, pointing out the raise in the brittleness of the cortical bone of the OVX + GLU rats. Treatment with BBL was statistically superior to FD and NBL treatment in increasing femoral midshaft peak load, stiffness, ultimate strength, and Young’s modulus. These perceptions provide evidence for the increase in measured mechanical characters including both the outside (cortical bone size and shape) and the inside bone characters (nature of the material properties of bone tissue). This can put down to the decreased bone resorption and/or the increased bone formation or both. Measuring the microarchitectural parameters, such as Tb.Sp, BS/BV, BMD, Tb.N, Tb.Th and BV/TV, may help us estimate the bone strength [38]. The OVX + GLU rats demonstrated a decrease in BMD, Tb.N, Tb.Th and BV/TV when compared with SHAM group. In addition, significantly higher levels of Tb.Sp and BS/BV were seen in PBS group when compared with SHAM group. It was discovered that treatment with BBL medicine prescription was statistically superior to other treatments in inhibiting the decrease of BV/TV and suppressing the increase of Tb.Sp. These parameters showed that BBL improved the trabecular organization and bone quality in the OVX + GLU rats. In histological analysis, we discovered that BBL strengthened the osteoblast activity and depressed the osteoclast function by up-regulating TB volume, as well as increasing cancellous bone mineralization rate and decreasing TRACP positive cells.

## Conclusions

We have successfully developed the novel biomineral-binding liposome formulation for the treatment of osteoporosis in the OVX + GLU rats. As the major formulation excipient, the pyrophosphate was conjugated to cholesterol and acted as the bone-binding moiety. The drug-containing liposome formulated with modified cholesterol demonstrated strong and fast binding capability to HA. When challenged with a disease model in rats of osteoporosis, the biomineral-binding liposome formulation of icariin demonstrated significantly better therapeutic efficacy than all the controls. Therefore, the application of BBL loaded with icariin can be a novel and effective candidate in future therapy of osteoporosis.

## Methods

### Materials

Icariin was purchased from Zelang (Nanjing, China; purity, 98%). Standard icariin was offered by Must BioTechnology Company (Chengdu, China; purity, ≥ 98%). Tris (tetra-*n*-butylammonium) hydrogen pyrophosphate (TBAP) was bought from Sigma-Aldrich Co. (St. Louis, MO). Soybean lecithin was got from A.V.T. Pharmaceutical Co. Ltd. (Shanghai, China). Cholesterol was got from solarbio Co. (Beijing, China). HA particles (DNA grade, Bio-Gel HTP gel) named as ‘synthetic HA’ in present study were got from Bio-Rad (Hercules, CA). The other reagents and solvents, if not appointed, were supplied by Kelong Chemical Reagent Factory (Chengdu, China).

The biomineral-binding lipid of PPi-TEG-Chol was synthesized as shown in Fig. 9 and the detail was shown in the Additional file 1.

**Fig. 9:** Synthesis of biomineral-binding material of PPi-TEG-Chol

### Preparation and characterization of liposomes

Liposomes were prepared by a combined method of a thin-film dispersion and a mechanical extrusion, including a main component of soybean lecithin (A), cholesterol (B), and PPi-TEG-Chol (C). The component ratio of BBL and NBL was optimized according to our previous report by central composite design that is widely used in designation of pharmaceutical dosage forms [39]. As shown in Table 1, to prepare BBL [A/B/C: 70/20/10 (molar ratios)] and NBL [A/B/C: 70/30/0 (molar ratios)], mixture of lipids and icariin was dissolved in 10 mL solvent of chloroform/methanol (1:1, v/v) and placed into a round bottom flask. The solvent was then removed under moderate vacuum until a thin film formed on the flask wall. The thin-film was further dried under vacuum condition for 24 h to confirm no chloroform left. Then the dried thin film was hydrated with phosphate-buffered solution (PBS, pH 7.4). Finally, the liposome suspensions were extruded through the 200-nm polycarbonate membrane in an Avanti^®^ Mini-Extruder to obtain the desirable size-dispersion liposomes. The empty biomineral-binding liposomes (EBBL) without icariin were prepared similarly except addition of icariin. Meanwhile, we prepared the fluore-labeled BBL (fluore-BBL) and fluore-labeled NBL (fluore-NBL) using sodium fluorescein to replace the aforementioned icariin in the preparation process.

Morphology of liposomes was observed under TEM on a JEM-100SX electron microscope (Japan). Particle size and the zeta potential of liposomes were characterized by DLS (Zetasizer Nano ZS90, Malvern Instruments, Malvern, UK).

Detections about encapsulation efficiency and drug-loading efficiency were conducted using an ultrafiltration tube with a molecular weight cut-off of 5 kDa (Solarbio Science and Technology Co., Ltd., Beijing, China). The un-encapsulated icariin (W_*free*_) was quantified using an Agilent 1260 HPLC system (Infinity, USA). Measurement was conducted on a reverse-phase C_18_ column (Agilent, 4.6 × 250 mm, 5 μm). The flow phase was a kind of mixture of acetonitrile and water (30:70, v/v) with a flow rate of 1.0 mL/min and an injection volume of 10 μL. Samples were diluted with methanol and filtered through a 0.22-μm membrane before injection. The detection wavelength was 270 nm. The selectivity, linearity, precision, and recovery of methods were fully validated. The encapsulation efficiency and the drug-loading efficiency were calculated using the following formula as: Encapsulation efficiency (%) = (W_*total*_ − W_*free*_)/W_*total*_ × 100%; Drug loading (%) = (W_*total*_ − W_*free*_)/W_*liposomes*_× 100%.

### HA rods’ synthesis and characterization

Because HA crystals are typically c-axis orientation on the surface of vertebrate long bone [33], to mimic the binding process of BBL with natural bone in vivo, we used a small intestinal submucosa (SIS) as the bio-template and prepared the plate-like single crystal HA with c-axis direction which was referred as ‘biotechnical HA’.

In the reaction system, the important key was the SIS, which acted as the bio-mineralization template. SIS was obtained according to the standard procedures [40]. Firstly, the tunica serosa and tunica muscularis of the fresh porcine small intestine should be removed, and SIS was washed with a saline solution. Secondly, SIS was immersed in solvent of methanol/chloroform (1:1, v/v) overnight in a fume hood, and the organic solvents were washed away with deionized water. Thirdly, SIS was kept in a mixed solvent of trypsin (0.05%) and ethylenediamine tetraacetic acid (0.05%) for overnight at 37 °C. Then saline solution was used to wash SIS to remove the trypsin and ethylenediamine tetraacetic acid. SIS was further treated with sodium dodecyl sulfate (0.5%) NaCl solution (0.9%). After shaking for 4 h, SIS was washed again with NaCl solution (0.9%). At last, SIS was immersed into a mixture of peroxyacetic acid (0.1%) and ethanol (20%) for 30 min, and further washed with NaCl solution (0.9%). The final product was freeze-dried and stored at 4 °C.

To prepare the experiment device as shown in Fig. 10, we made a hole in the middle of the cap of a centrifuge tube (50 mL) and sealed it with SIS membrane. Then, a solution of K_2_HPO_4_ (30 mL, 0.1 M) was added into it. This tube was inverted and soaked into a beaker filled with solution of Ca(CH_3_COO)_2_ (30 mL, 0.1 M). This reaction system imitating the bone mineralization conditions was incubated for 7 days (37 °C, pH 7.4). Finally,the morphology and structure of HA rods were analyzed using a scanning electron microscopy.

**Fig. 10:** Preparation and characterization of the biotechnical HA. The whole self-design device (**a**) was kept in a constant-temperature incubator at 37 °C. The SIS covered the hole in the middle of the tube cap. The top surface of SIS membrane continuously touched with K_2_HPO_4_ solution and the lower one contacted with Ca(AC)_2_ solution. After the crystal formed on the bottom surface of SIS membrane, the whole SIS membrane was peeled off and subjected to analyze the morphology and structure using scanning electron microscopy of FEI Inspect F50 (**b**)

### Binding ability and kinetics of BBL on the synthetic and biotechnical HA particles

The fluorescein sodium-loaded liposomes including fluore-BBL and fluore-NBL were prepared using the method described above. For the binding ability experiment, both the commercial synthetic HA and the biotechnical HA produced by bio-template SIS were added into the fluorescein sodium-loaded liposomal solutions. The mixtures were agitated for half an hour at room temperature. Further, it was filtered, washed with water, and lyophilized. Finally, HA particles were observed under a fluorescence microscope. For the binding kinetics experiment, these two types of HA (100 mg) were added into 1.0 mL of icariin-loaded liposomal solutions. HA was eliminated by centrifugation (10,000×*g*, 5 min) after incubation for 1, 3, 5, 10, 30 min respectively at room temperature. The supernatant was collected and the content of icariin left in liposomal supernatant (W_*left*_) after binding was analyzed by HPLC method mentioned above. Binding rate (%) was calculated according to the following formula as: Binding rate (%) = (W_*total*_ − W_*left*_)/W_*total*_× 100%. NBL without PPi-TEG-Chol were used as control in the experiment.

### In vitro icariin release study of BBL

The in vitro release analysis of icariin from liposomes was conducted in PBS medium (10 mM, pH 7.4). Liposomal formulations and free icariin were put into a dialysis bag (MWCO, 3 kDa) placed in 30 mL of release medium with gentle stirring at 37 °C. At pre-designed time intervals, 1.0 mL of samples were taken out from the release medium and replaced with fresh medium. Every group of sample was diluted to 2.0 mL and filtered through a 0.22-μm membrane (Millipore). Amount of icariin in all samples was determined using HPLC method as mentioned above.

### Ovariectoporosis model

All Sprague–Dawley (SD) rats obtained from the Laboratory Animal Center of Southwest Medical University were maintained at 20–25 °C under a 12-h light/dark cycle and allowed for food and water. All animal experiments were approved by the Animal Ethics Committee of Southwest Medical University (Permit No. 20160126). The animal handling and surgical procedures were carried out in accordance with the guidelines of the Local Animal Use and Care Committees of Lu Zhou.

For establishing the osteoporosis model, 3-month-old mature female SD rats were subjected to bilateral OVX or sham-control surgery (SHAM) according to the Ref. [25]. Briefly, rats were anesthetized by intraperitoneal injection of sodium pentobarbital (1%, 8 mL/kg). The back fur of rats was shaved, cleaned with iodophor solution, and then covered with a sterile cloth. A single longitudinal lumbar lateral skin incision was made near the midpoint of lower edge of free ribs and iliac crest, where the ovary was located. Before removing the ovary, a suture was put in around the ovarian artery and vein to ligate the ovary. The muscles were repositioned in layers and sutured with re-absorbable sutures. The skin incision was closed using nylon 4-0 sutures. OVX rats were injected intraperitoneally with dexamethasone (a synthetic GLU, 0.5 mg/kg) twice a week for 4 weeks. The rats in SHAM group were subjected to SHAM surgery, in which the ovaries were exposed but kept intact. The bone mineral density (BMD) of bilateral femur was measured using micro-CT (SIMENS healthcare, Berlin and Munich, Germany) at 7 weeks post surgery, respectively. The rats were divided into six groups (n = 8) following as: SHAM, PBS as control, NBL, free drug (FD) and BBL. The animals were treated with or without icariin as mentioned above on every day by intraperitoneal injection, in which the formulations were normalized to the amount of icariin (90 mg/kg), and FD was prepared by dissolving icariin into PEG 400 (0.2%) and further being diluted with saline for injection. Seven weeks post-treatment, animals were anesthetized and blood was collected and subjected to detection for the bone formation marker of ALP and bone resorption marker of TRACP 5b. The bilateral femoral bones were extracted for bone biomechanical examination, Micro-CT scanning, and histology analysis.

### Serum biochemical analysis

The bone formation was assessed by measuring serum level of ALP and the bone resorption was evaluated by measuring serum level of TRACP 5b. Measurements of serum ALP and TRACP 5b were performed by a sandwich enzyme-linked immunosorbent assay (ELISA, Qiao Du Biotechnology Co., Ltd. Shanghai, China) according to the protocols offered by provider. Briefly, the standards and samples were added into the standard wells and the sample wells, respectively. Then horseradish peroxidase (HRP) were added to each well, and the mixture were incubated for 60 min at 37 °C. After rinse with washing solution for 5 times, a chromogen solution were added to each well and mixed gently. The mixture was incubated for another 15 min in the dark at 37 °C. At last, a stopping solution was added to each well to end the reaction, and then optical density was measured at 450 nm using a microplate reader within 15 min.

### Bone biomechanical examination

Mechanical characteristics of femur from the treated rats were evaluated by a three-point bending test using a universal testing machine (Jinan Huaxing Test Equipment Co., Ltd. ShanDong, China). Prior to test, the bones were balanced to room temperature and kept moist until the test was finished. The length of bone was obtained using a caliper. The femur was placed on the holding device with supports located apart 12 mm from each other. A bending force was applied to the cross head at a speed of 0.033 mm/s until the femur fractured. According to the experimental data, the load–displacement curve can be plotted for each sample. Some mechanical characteristics were obtained from these curves, including peak load (the maximum force that the bone withstood before fracture), ultimate stiffness (the extrinsic rigidity of femur before fracture), ultimate strength (the maximum stress of femur before fracture) and the Young’s modulus representing the intrinsic stiffness of an intact bone.

### Micro-CT analysis

To evaluate skeletal microarchitecture, the right femora (n = 6) were subjected to a high-resolution Micro-CT analysis using a Micro-CT imaging system (Siemens, Inveon), according to the method described in a publication [41].

The quantitative parameters of the bone microstructure were measured, including BV/TV, BS/BV, Tb.Th, Tb.N, Tb.Sp and BMD. All the digitalized data and 3-dimensional images were supplied by the built-in software of Micro-CT (Siemens, Inveon).

### Histological analysis

In order to assess the bone mineral areas, femora were fixed in 4% paraformaldehyde, decalcified with EDTA (10%, pH 7.4), and embedded using paraffin. Longitudinal serial sections (6 μm) were mounted on polylysine-coated microscope slides. For general histological studies, H&E staining, TRACP staining, and Alizarin Red staining were performed according to manufacturer’s protocol. The stained areas were quantified by ImageJ software.

### Statistical analysis

All data are expressed as mean ± SD after at least three separate tests. The differences among the treatment groups were analyzed for significance using the Student t-test. A *P* value less than 0.05 was regarded as statistical significance and a higher significance level was set at *P *< 0.01.

## Additional file

**Additional file 1.** Synthesis of biomineral-binding lipid of PPi-TEG-Chol and pharmacokinetics evaluation of BBL in Rats. **Figure S1.** Mean plasma concentration-time profile of icariin in rats after intraperitoneal administration. **Figures S2–S5.** ^1^H NMR spectra of synthetic products.

## Abbreviations

ALN-TEG-Chol: alendronate-tri(ethyleneglycol)-cholesterol
ALP: alkaline phosphatase
BBL: biomineral-binding liposomes
BMD: bone mineral density
BMP-2: bone morphogenic protein-2
BS/BV: bone surface per bone volume
BV/TV: bone volume per tissue volume
CCD: central composite design
DCC: *N*,*N*′-dicyclohexylcarbodiimide
DCM: dichloromethane
DLS: dynamic light scattering
DMAP: 4-dimethylaminopyridine
EBBL: empty biomineral-binding liposomes
ELISA: enzyme-linked immunosorbent assay
FD: free drug
GLU: glucocorticoid
GRAS: Generally Regarded As Safe
HA: hydroxyapatite
H&E: hematoxylin and eosin
HRP: horseradish peroxidase
Micro-CT: micro-computerized tomography
NBL: non-binding liposome
OVX: ovariectomy
PBS: phosphate-buffered saline
PDI: polydispersity index
PPi: pyrophosphate ions
PPi-TEG-Chol: pyrophosphate-tri(ethyleneglycol)-cholesterol
SD: Sprague–Dawley
SHAM: sham-control surgery
SIS: small intestinal submucosa
TB: trabecular bone
Tb.N: trabecular number
Tb.Sp: trabecular separation
Tb.Th: trabecular thickness
TBAP: tris (tetra-*n*-butylammonium) hydrogen pyrophosphate
TEM: transmission electron microscopy
TRACP 5b: tartrate-resistant acid phosphatase 5b
